# The Preventive Effects of Naringin and Naringenin against Paclitaxel-Induced Nephrotoxicity and Cardiotoxicity in Male Wistar Rats

**DOI:** 10.1155/2022/8739815

**Published:** 2022-09-30

**Authors:** Shimaa S. Khaled, Hanan A. Soliman, Mohammed Abdel-Gabbar, Noha A. Ahmed, Kandil Abdel Hai Ali Attia, Hesham A. Mahran, El-Shaymaa El-Nahass, Osama M. Ahmed

**Affiliations:** ^1^Biochemistry Department, Faculty of Science, Beni-Suef University, P.O. Box 62521, Beni-Suef, Egypt; ^2^Physiology Division, Zoology Department, Faculty of Science, Beni-Suef University, P.O. Box 62521, Beni-Suef, Egypt; ^3^Clinical Nutrition Department, College of Applied Medical Sciences, Jazan University, P.O. Box 114, Jazan 45142, Saudi Arabia; ^4^Health Informatics Department, College of Public Health & Tropical Medicine, Jazan University, P.O. Box 114, Jazan 45142, Saudi Arabia; ^5^Hygiene, Zoonosis and Epidemiology Department, Faculty of Veterinary Medicine, Beni-Suef University, Beni-Suef, Egypt; ^6^Department of Pathology, Faculty of Veterinary Medicine, Beni-Suef University, P.O. Box 62521, Beni-Suef, Egypt

## Abstract

This study assessed the preventive properties of naringin and naringenin on paclitaxel-induced nephrotoxicity and cardiotoxicity in adult male Wistar rats. Intraperitoneal injection of paclitaxel 2 mg/kg body weight, two days/week on the 2nd and 5th days of each week, with or without oral administration of naringin and/or naringenin 10 mg/kg body weight every other day, was continued for six weeks. Treatment of rats with naringin and/or naringenin significantly reversed elevated serum creatinine, urea, and uric acid levels caused by paclitaxel, reflecting improved kidney function. Similarly, heart dysfunction induced by paclitaxel was alleviated after treatment with naringin and/or naringenin, as evidenced by significant decreases in elevated CK-MB and LDH activities. After drug administration, histopathological findings and lesion scores in the kidneys and heart were markedly decreased by naringin and/or naringenin. Moreover, the treatments reversed renal and cardiac lipid peroxidation and the negative impacts on antioxidant defenses via raising GSH, SOD, and GPx. The preventive effects of naringin and naringenin were associated with suppressing oxidative stress and reestablishing antioxidant defenses. A combination of naringin and naringenin was the most efficacious in rescuing organ function and structure.

## 1. Introduction

Paclitaxel is a natural tricyclic diterpenoid isolated from the bark of *Taxus brevifolia* (Pacific yew). The chemical is a taxane, an intermediary metabolite that displays potent anticancer activity [1–3]. Taxanes are used for treating different forms of cancer and are initial therapy for earlier stages of these diseases [4–7]. Moreover, paclitaxel is recognized worldwide as the number one chemotherapeutic agent [8]. Paclitaxel is used in the treatment of aggressive and metastatic breast cancer, ovarian cancer, lung cancer, pancreatic cancer, and many other malignancies [9]. Unfortunately, paclitaxel is poorly soluble in water and other solvents for the formulation of injectables and causes serious side effects, such as hypersensitivity, neutropenia, myelosis, neutropenia, and neurotoxicity [10].

A paclitaxel formulation using Cremophor EL (CrEL) as a solvent (Taxol) induced cumulative sensory-dominant peripheral nephrotoxicity in humans, clinically characterized by numbness and paresthesia of the extremities. This toxicity was a result of CrEL exposure. Serum creatinine levels increased in association with increased damage [11–15]. Additionally, paclitaxel caused cardiac complications, especially conduction blocks, sinus bradycardia, bradycardia, ventricular tachycardia, and ischemic manifestations [16, 17].

Paclitaxel produces cytotoxicity by enhancing the formation of reactive oxygen species (ROS), thus inducing oxidative stress [18, 19]. Hence, a search for natural chemicals that augment the antitumor activity of paclitaxel or moderate its toxicity, such as flavonoids and polyphenols, are attractive alternatives [20–23].

Natural therapeutics have been investigated to prevent the side effects of anticancer drugs [24–28], highlighting the relevance of medicinal herbs and their bioactive constituents [29–32]. Moreover, phytochemicals may prove clinically useful for improving treatment efficacy for cancer patients and reducing the incidence of adverse reactions [33]. Flavonoids are phytochemicals that inhibit the growth of tumor cells *in vitro* and *in vivo* [34]. Flavonoids exhibit several biological properties, including antioxidant, antimutagen, anticancer, antibacterial, and anti-inflammatory [35]. Naringin and naringenin are citrus flavonoids with pharmacological properties, especially antioxidant, antifree radical, anti-inflammatory, and blood lipid reduction [36]. Additionally, naringin and naringenin are potent anticancer agents and play a role in the management of various tumors [37].

Concerning previous studies, using plant constituents with antioxidant and anti-inflammatory properties will be our strategy to counteract and treat the side effects of anticancer drugs. As a result, this investigation was carried out to assess the renal and cardiac toxicity prevention by naringin and naringenin coincident with paclitaxel-treated Wistar rats. We assessed toxicity by examining kidney and heart function, oxidative stress, and antioxidant defense systems, as well as histopathology.

## 2. Materials and Methods

### 2.1. Experimental Animals

Fifty adult male Wistar rats with weights of ∼130–150 g were collected from the VACSERA Vaccination Centers' Animal House in Dokki, Giza, Egypt. In order to rule out any concurrent infections, animals were watched for 15 days before the experiment began. Rats were housed in polypropylene cages with ventilated stainless steel lids at a standard air temperature of (25 ± 5°C) and with a 12-hour light cycle. Animals had free access to water and received a sufficiently balanced standard diet on a daily basis *ad libitum*. All animal-related procedures were performed, complying with the recommendations and instructions of the Experimental Animal Ethics Committee, Faculty of Science, Beni-Suef University, Egypt (Ethical Approval Number: BSU/FS/2017/7.) We did everything we could to lessen animals' pain and suffering.

### 2.2. Chemicals

Paclitaxel (Taxol®) was obtained from the Bristol–Myers Squibb global biopharmaceutical company (batch code: 7E05628). Naringin (batch code: BCBM4171 V) and naringenin (batch code: BCBJ2179 V) were obtained from Sigma (MO, USA). The creatinine reagent kit (catalog numbers: M11502c-18) and the urea reagent kit (catalog numbers: M11536c-16) were purchased from Biosystem S.A. (Spain). Uric acid, CK-MB, and LDH reagent kits were purchased from Spin React (Spain), with catalog numbers MD41001, MD41254, and MX41214, respectively. Chemicals of oxidative stress including trichloroacetic acid were obtained from PanReac AppliChem ITW Companies (Spain) (batch code: 5O011689), thiobarbituric acid was obtained from Sd Fine Chem Limited(SDFCL) Company (India) (batch code: *L* 16 A/1916/1212/13), 1,1,3,3 tetra-methoxy propane was obtained from Sigma-Aldrich (MO, USA) (catalog no: T9889), metaphosphoric acid was obtained from ALPHA CHEMIKA Company (India) (batch code: M 21519), 5,5- dithiobis nitrobenzoic acid was obtained from Sigma-Aldrich (MO, USA) (batch code: 40K3652), GSH was obtained from PanReac AppliChem ITW Companies (Spain) (batch code: 3W010085), and pyrogallol was obtained from Research Lab Company (India) (batch code: 1280B251114).

### 2.3. Experimental Design

In this study, adult male Wistar rats were divided into five groups, each with ten rats.

1. Normal group: rats were administered 5 mL 1% carboxymethyl cellulose (CMC) kg body weight (b.wt) orally every other day and 2 mL saline twice per week intraperitoneally for six weeks.
2. Paclitaxel-administered control group: rats were administered paclitaxel intraperitoneally at a dose level of 2 mg/kg b.wt [38] twice weekly on the 2nd and 5th days of each week. This group was also given the corresponding amount of 1% CMC (5 mL/kg b.wt) orally every other day for six weeks.
3. Paclitaxel-administered group treated with naringin: rats were administered paclitaxel intraperitoneally as in group 2 and received oral naringin 10 mg/kg b.wt treatment [39] every other day for six weeks (dismantled in 5 mL 1% CMC).
4. Paclitaxel-administered group treated with naringenin: rats were treated as above but were administered naringenin at a dose level 10 mg/kg b.wt [40] (dismantled in 5 mL 1% CMC) instead of naringin every other day for six weeks.
5. Paclitaxel-administered group treated with a combination of naringin and naringenin: rats were treated as above but received both naringin and naringenin at dose levels of 10 mg/kg (dismantled in 5 mL 1% CMC) b.wt every other day for six weeks.

### 2.4. Collection of Blood and Tissue Samples

Using diethyl ether inhalation anesthesia before decapitation and dissection and at the end of the experiment, blood samples were taken from each animal's jugular vein into gel and clot activator tubes, allowed to coagulate at room temperature, and then centrifuged at 3,000 rpm for 15 min. Clearly, nonhemolyzed sera were aspirated quickly, divided into four aliquots, and kept at 30°C until they were needed for biochemical testing. Each animal's kidney and heart tissues were rapidly removed and weighed after decapitation and dissection. A portion of tissue of each organ was preserved in phosphate-buffered formalin (10%) for 24 h before being transferred to 70% alcohol for histological analysis. About 0.5 g of each tissue was homogenized in 5 mL saline (0.9% NaCl) with a Teflon homogenizer (Glas-Col, Terre Haute, USA). After the homogenates had been centrifuged for 15 minutes at 3,000 rpm, the supernatants were aspirated from the homogenates and kept in a deep freezer at −20°C for determination of oxidative/antioxidant status.

### 2.5. Examination of Serum Biomarkers for Kidney Function

Creatinine and urea levels in serum were measured as previously described by Fabiny and Ertingshausen [41] and Tabacco et al. [42]. Uric acid was assessed using the method of Fossati et al. [43].

### 2.6. Examination of Serum Biomarkers for Heart Function

CK-MB and LDH activities in serum were assayed as described by Young [44] and Young [45].

### 2.7. Assessment of Kidney and Heart Oxidative Stress and Antioxidant Levels

Kidney and heart lipid peroxidation (LPO) was estimated as previously described by Preuss et al. [46]. Briefly, protein was precipitated by adding 75 *μ*L of 76% trichloroacetic acid (TCA) to 0.5 mL of the kidney or heart homogenate. Then, 175 *μ*L of 1.07% thiobarbituric acid (TBA) was added. After 30 minutes in a water bath at 80°C, the formed faint pink color was detected at 532 nm. The standard was MDA (malondialdehyde or 1,1,3,3-tetramethoxypropane).

Kidney and heart GSH content was estimated by following the findings reported by Beutler et al. [47] with modifications by the addition of 0.5 mL 5,5′-dithiobis (2-nitrobenzoic acid) or Ellman's reagent for color development and phosphate buffer solution (pH 7) to homogenate supernatants after protein precipitation. The generated yellow color in samples and GSH standards were quantified at 412 nm against blank.

Kidney and heart glutathione peroxidase (GPx) activity was measured as previously described by Matkovics et al. [48]. This method is based on detecting GSH that has been transformed into oxidized glutathione (GSSG) through the detection of residual GSH and deducting it from the total. Briefly, 50 *μ*L of the homogeneous supernatant was placed in a Wasserman tube containing 350 *μ*L Tris buffer (pH 7.6), 50 *μ*L GSH solution (2 mM), and 50 *μ*L H2O2 (3.38 mM). The residual GSH content was determined after a 10-minute incubation period, as indicated previously. A standard was made by substituting 50 *μ*L distilled water for 50 *μ*L of the sample, and a blank was made by substituting 100 *μ*L distilled water for 50 *μ*L of the sample and 50 *μ*L GSH solution. The amount of GSH transformed to GSSG was then determined using the residual GSH content, and the enzyme activity was calculated.

The activity of superoxide dismutase (SOD) in the kidney and the heart was measured as previously described by Marklund and Marklund [49]. The procedure is focused on the suppression of auto-oxidation of pyrogallol by SOD. The presence of superoxide ions is required for the process to work. One unit of enzyme activity is the amount of an enzyme that reduces extinction by 50% in one minute relative to the control.

### 2.8. Histopathological Examination

Parts of the kidneys and hearts of rats were collected and fixed in 10% neutral buffered formalin for 24 h. Tissues were then washed with water and dehydrated in a series of ethyl alcohol dilutions (50%, 70%, 90%, 95%, 100%). Specimens were cleaned with xylene before being embedded in paraffin wax for 24 hours at 56°C in a furnace. Four *μ*m sections were cut from paraffin wax tissue blocks with a sliding microtome. For regular examination under an electric light microscope, the tissue sections were fixed on glass slides, dewaxed, and hematoxylin and eosin stained (H&E) [50]. Histopathological lesion scores were identified as previously described by El-Far et al. [51]. Score scale: 0 = normal; + ≤ 25%; ++ = 26–50%; +++ = 51–75%; ++++ = 76–100%. The lesions were graded in a blinded manner.

### 2.9. Statistical Analysis

All data were presented as the mean ± standard error of the mean (SEM). For statistical analysis, Statistical Package for the Social Sciences (SPSS) programme (version 22) (IBM software, USA) was utilized. Tukey's post hoc test was used to compare mean values pairwise. Differences were deemed significant at *p* < 0.05.

## 3. Results

### 3.1. Effect of Treatments on Kidney Function Parameters in Serum

Administration of paclitaxel to rats for 6 weeks produced a significant increase (*p* < 0.05) in serum urea, creatinine, and uric acid levels. Percentage changes were +52.43, +106.98, and +352.46%, respectively, compared to normal controls.

The increased urea, creatinine, and uric acid levels in paclitaxel-administered rats were significantly reduced after treatment with naringin and the combination. However, treatment with naringenin produced significant decreases only in elevated creatinine and urea levels; uric acid levels decreased but not significantly (*p* > 0.05). The naringin and naringenin combination seemed to be the most efficacious for normalizing elevated serum levels. Percentage decreases in urea, creatinine, and uric acid were −28.75, −47.19, and −40.22%, respectively, compared with paclitaxel alone (Table 1).


(1) $$\begin{array}{c} \text{\%change}=\left(\frac{\text{Final value}–\text{Initial value}}{\text{Initial value}}\right)\times 100\left[52\right]. \end{array}$$

### 3.2. Effect of Treatments on Heart Function Biomarkers in Serum

Administration of paclitaxel to rats for 6 weeks stimulated a significant rise in serum CK-MB and LDH activities with percentage changes of +359.26 and + 293.55%, respectively, in comparison to the normal control group. The treatment of paclitaxel-administered rats with naringin and naringenin and their combination produced significant decreases in the elevated CK-MB activity with percentage changes of **−**46.13, **−**55.52, and **−**47.76%, respectively. Similarly, LDH activity also significantly decreased after treatment with naringin and naringenin and their combination recording percentage decreases of **−**46.41, **−**48.86, and **−**50.81%, respectively (Table 2).


(2) $$\begin{array}{c} \%\text{change}=\frac{\text{Final value}–\text{ Initial value}}{\text{Initial value}}\times 100\left[52\right]. \end{array}$$

### 3.3. Effect of Treatments on the Parameters of Antioxidant Defence and Oxidative Stress in the Kidneys and the Heart

As outlined in Table 3, administration of paclitaxel to rats significantly raised kidney LPO (+54.93%) and significantly decreased GSH levels (**−**53.09%) and SOD (**−**8.19%) and GPx (**−**23.23%) activities in comparison to the normal control group. The oral dose of naringin and naringenin and their combination improved kidney LPO significantly. Additionally, treatment with naringin and naringenin or their combination resulted in a significant increase in kidney GSH content. Also, these treatments reversed the decline in activities of kidney SOD and GPx.


(3) $$\begin{array}{c} \text{\%change}=\frac{\text{Final value }–\text{Initial value}}{\text{Initial value}}\times 100\left[52\right]. \end{array}$$

In a similar way as in the kidney, paclitaxel administration resulted in a significant increase in LPO in heart tissue, whereas heart GSH content, SOD activity, and GPx activity decreased significantly. Naringin and naringenin and their combination significantly increased cardiac LPO. Additionally, heart GSH content was significantly increased as a result of the treatment with naringin and the combination. However, the treatment with naringenin resulted in a nonsignificant rise in heart GSH content. Moreover, all three treatments significantly enhanced heart SOD and GPx activities (Table 4).


(4) $$\begin{array}{c} \%\text{change}=\frac{\text{Final value}–\text{ Initial value}}{\text{Initial value}}\times 100\left[52\right]. \end{array}$$

### 3.4. Kidney Histopathology

Renal lesions are illustrated in Table 5 and Figure 1. Histological examination of kidney sections of normal control rats exhibited normal histological construction (Figure 1(a)). Conversely, paclitaxel administration resulted in deleterious histological changes and a variety of lesions, including severe lesions, mostly in the form of severe mononuclear leukocyte inflammatory cell infiltration, degenerative changes combined with nuclear pyknosis of the renal lining epithelium, and apoptosis (Figures 1(b) and 1(c)). The apoptotic morphological changes include cell shrinkage, nuclear shrinkage, hypereosinophilic cytoplasm due to cytoplasmic condensation, nuclear condensation, nuclear fragmentation (karyorrhexis), nuclear pyknosis, apoptotic blebs, and rounded hyperchromatic apoptotic bodies. Severe glomerulonephritis was also observed. Additionally, there was focal interstitial nephritis that was escorted by glomerular tuft and interstitial blood capillary congestion (Figure 1(b)). When rats receiving paclitaxel were given naringin, some histological changes and a number of lesions were observed, such as the degeneration and necrosis of the renal lining epithelium and focal mononuclear leukocyte inflammatory cells in interstitial tissues, which were accompanied by mild glomerulonephritis and mild apoptosis (Figure 1(d)). Paclitaxel/naringenin-treated rats exhibited milder lesions than paclitaxel/naringin- treated rats (Figure 1(e)). The administration of paclitaxel/naringin/naringenin showed a quite improvement in renal lesions compared to other treated rats (Figure 1(f)).

### 3.5. Heart Histopathology

Cardiac pathological lesions are described in Table 6 and Figure 2. Intact histological structures in cardiac muscles were observed in tissues from normal controls (Figure 2(a)). The paclitaxel administration produced many heart histological deleterious changes, including severe degenerative changes and necrosis of cardiac muscles, as well as mild apoptotic changes (AP) represented by apoptotic cells characterized by condensed eosinophilic cytoplasm and condensed pyknotic nuclei (Figure 2(b)). Also, minimal apoptotic changes are shown in Figure 2(c). Treatment with naringin (Figure 2(d)), naringenin (Figure 2(e)), and their combination (Figure 2(f)) produced notable reversal of paclitaxel-induced histological changes.

## 4. Discussion

Paclitaxel is largely effective for ancillary treatment of tumors in ovarian [53] and breast cancer [54, 55]. Unfortunately, paclitaxel therapy can increase acquired resistance, resulting in chemotherapy failure [56]. Further, paclitaxel has limited clinical application due to its low water solubility and low compatibility with excipients in formulations [5]. Paclitaxel raised levels of oxidative and nitrosative stress markers in mice [57] and may have caused kidney damage due to ROS generation, which induces oxidative stress [58]. Moreover, paclitaxel induces oxidative stress and cardiotoxicity in adult male Wistar rats [59].

The current study showed the impact of serial intraperitoneal injections of paclitaxel over a period of six weeks at the dose level of 2 mg/kg b.wt 2 days/week. These injections induced nephrotoxicity evidenced biochemically by a significant elevation of serum urea, creatinine, and uric acid levels. Thus, the drug impairs renal function and may compromise urinary excretion of toxic metabolites. Our data are consistent with those reported by Adikwu et al. [58]. Ahmed et al. [60] also found that paclitaxel affected renal function, reflected in significant elevation of serum urea and creatinine levels in adult male albino rats. In the current investigation, histopathological analysis of renal sections of paclitaxel-administered rats supported the previous biochemical results. The kidney exhibited several adverse histological changes and lesions, including severe degenerative changes in renal epithelium associated with focal lymphocytic infiltration and severe glomerulonephritis. Moreover, focal interstitial nephritis and moderate apoptotic lesions were observed, accompanied by congestion in interstitial blood capillaries and the glomerular tuft. Previous studies indicated that paclitaxel treatment causes congested glomerular capillaries, cellular infiltration, extravasation, and vacuolated tubular cells [60]. Similarly, Choudhury et al. [61] observed atrophic changes in glomeruli and kidney tubules in experimental animals treated with paclitaxel, which may be due to high CrEL content. Paclitaxel also adversely affected renal morphology by inducing hypercellular glomeruli and tubular necrosis combined with apoptotic changes [58,62]. Apoptosis is mediated by caspases, a family of cysteine proteases whose stimulation is triggered by specific apoptotic stimuli and whose substrates include numerous proteins [63], and the restricted cleavage of which results in apoptosis-like morphological features [62].

Citrus flavonoids naringin and naringenin have anti-inflammatory and antioxidant effects both *in vivo* and *in vitro* [64]. In comparison to many previous studies, natural products offer the best hope for improving tumor-targeting drugs [65–69]. In our study, treatment of paclitaxel-administered rats with naringin and naringenin or their combination reduced elevated urea, creatinine, and uric acid levels and substantially restored histological integrity in agreement with previous studies by Ahmed et al. [70] who reported that naringin and naringenin enhanced kidney function and structural integrity in male rats. Also, naringin countered nephrotoxicity induced by methotrexate in male rats [71], and naringenin was nephroprotective against carbon tetrachloride-induced nephrotoxicity in mice [72]. Quercetin, a similar flavonoid, has been shown to alleviate renal and pancreatic tissue alterations caused by D-galactose in rats [51].

In the present study, paclitaxel administration also induced cardiotoxicity, evidenced biochemically by a significant increase in serum activity of CK-MB and LDH. Histopathological findings supported these changes in serum enzyme activities. The hearts of the paclitaxel-administered group exhibited several adverse histological changes and lesions, including severe degenerative changes and necrosis of cardiac muscles accompanied by the presence of inflammatory and apoptotic cells. These findings concur with those of Saad et al. [73] who indicated that paclitaxel treatment resulted in a marked increase in serum activities of (LDH and CK-MB) and also produced cytoplasmic vacuolation of heart myocytes. Additionally, Malekinejad et al. [59] found that paclitaxel increased CK-BM activity and produced pathological lesions, such as diffuse edema, hemorrhage, hyaline exudates, congestion, and necrosis. Moreover, increased LDH activities in patients treated with paclitaxel are associated with oxidative prehemolytic injury, as observed previously *in vitro* [74]. Besides, paclitaxel treatment affects adult cardiomyocytes, mainly noticeable in changes in myofibrillar structure and function [75]. Paclitaxel was also reported to induce apoptosis in cardiac tissue [76].

In the current study, treatment of paclitaxel-administered rats with naringin and/or naringenin resulted in improvement in cardiac biomarkers and histological integrity. These outcomes are in line with those of Rajadurai and Prince [77] who showed that naringin improved cardiac biochemical and histopathological alterations induced by isoproterenol in Wistar rats. The agent also protects against cardiac toxicity induced by doxorubicin *in vivo* and *in vitro* [78–80]. Moreover, Zhao et al. [81] reported that naringenin protects the cardiovascular system from palmitate-induced apoptosis in endothelial cells of human umbilical veins.

Renal and cardiac toxicity in paclitaxel-administered rats was correlated with a noticeable rise in kidney and heart LPO and a reduction in nonenzymatic antioxidant GSH content and enzymatic antioxidant (SOD and GPx) activities. These findings corroborate the findings of several other researchers [82–84] who reported that paclitaxel treatment weakens antioxidant defense systems. Paclitaxel administration caused renal damage *via* ROS generation, resulting in oxidative stress [58, 85]. Also, strong evidence exists that oxidative stress is closely associated with cardiotoxicity induced by antitumor drugs [86]. Moreover, administration of paclitaxel caused a notable increase in LPO as well as an increase in NO levels in the heart [59].

The current study's findings showed that administering naringin and/or naringenin decreases LPO, increases GSH content, and augments SOD and GPx activities in kidney and heart tissue after six weeks of treatment. This improvement may be attributed to scavenging ROS and free radicals induced by paclitaxel intoxication. These findings are consistent with those of the research by Fukui et al. [87] who proved that flavonoids inhibit paclitaxel-induced ROS generation. Moreover, Cavia-Saiz et al. [88] showed that naringin and naringenin are potent free radical scavengers and can prevent LPO. Harisa [89] proposed that naringin reversed paclitaxel-induced erythrocyte aging by reducing oxidative stress. Also, Sahu et al. [90] suggested that naringenin restored antioxidant enzymes by scavenging free radicals *via* its OH group and that this scavenging was responsible for reduced hepatic and renal damage.

## 5. Conclusion

Naringin and naringenin and their combination prevent many adverse impacts on renal and cardiac function and histological integrity induced by paclitaxel in Wistar rats. This action is due to suppressing oxidative stress and enhancing antioxidant defense systems in both organs. The combination of naringin and naringenin was the most efficacious for protecting kidney and heart function and structural integrity. An important limitation of the study is the shortage of kidney and heart samples to perform Western blot analysis for determination of various mediators of apoptosis and inflammations due to their exhaustion in detection of oxidative stress/antioxidants biomarkers and histological investigations. Furthermore, clinical studies are required to assess the safety and efficacy of naringin and naringenin and their combination against paclitaxel-deteriorated effects on the heart and kidneys in human beings.

## Figures and Tables

**Figure 1:** Photomicrographs of kidney sections of different experimental groups. **(a)** A photomicrograph of a kidney segment of healthy rats revealed glomeruli (G), proximal tubules (PTs), and distal tubules (DTs) and all had typical histologic structures. **(b)** A photomicrograph of the kidney section of paclitaxel-administered rats passing through the blood vessel (BV) underwent significant degenerative changes (DCs) that were linked with localized mononuclear leukocyte infiltration (IC). **(c)** Another kidney section of paclitaxel-administered rats revealed the presence of severe apoptotic changes (AP). **(d**) A photomicrograph of the kidney section of rats given paclitaxel and treated with naringin revealed mild apoptotic changes (AP) and mild degenerative changes (DCs) linked with lymphocytic infiltration (IC). (**e)** A photomicrograph of the kidney section of rats given paclitaxel and treated with naringenin showing congested glomerulus (CG), mild degenerative changes (DCs), minor apoptotic changes (AP), focal pyknotic nuclei (PN), and significant inflammatory cell infiltration were all visible (IC). **(f)** A kidney section of rats given paclitaxel and treated with a combination of naringin and naringenin showing infiltration of inflammatory cells (ICs), minor apoptotic changes (AP), and minor degenerative changes (DCs) (H&E; 400X).

**Figure 2:** Photomicrographs of heart sections of different experimental groups. (a) A section of the rat's normal heart was photographed, revealing the typical histologic anatomy of its cardiac muscles (CM). (b, c) The heart of a paclitaxel-treated rat is shown in a photomicrograph, with marked degenerative changes (DCs), inflammatory cell infiltration (IC), hyalinosis (H), and apoptotic changes (AP). (d) The cardiac tissue of rats given paclitaxel and naringin revealed moderate degenerative changes (DCs) and minor apoptotic changes (AP). (e) Mild hyalinosis (H) was visible in the cardiac section of paclitaxel-administered rats treated with naringenin. (f) A section of the heart of paclitaxel-administered rats treated with a combination of naringin and naringenin revealed moderate degenerative changes (DCs) linked with minimal inflammatory cell infiltration (IC) (H&E; 400X).

**Table 1:** Effect of naringin and/or naringenin on serum parameters related to kidney function.

Parameters and groups	Creatinine (mg/dl)	% change	Urea (mg/dl)	% change	Uric acid mg/dl	% change
Normal	0.43 ± 0.04	**—**	26.70 ± 1.17	**—**	0.61 ± 0.09	**—**
Paclitaxel	0.89 ± 0.04^a^	106.98	40.70 ± 1.98^a^	52.43	2.67 ± 0.29^a^	352.46
Paclitaxel + naringin	0.65 ± 0.05^ab^	**−**26.97	29.20 ± 1.66^b^	**−**28.26	1.72 ± 0.13^ab^	**−**37.68
Paclitaxel + naringenin	0.53 ± 0.04^b^	**−**40.45	30.80 ± 1.08^b^	**−**24.32	2.22 ± 0.79^a^	**−**19.57
Paclitaxel + naringin + naringenin	0.47 ± 0.02^b^	**−**47.19	29.00 ± 1.37^b^	**−**28.75	1.65 ± 0.08^ab^	**−**40.22

Data are expressed as mean ± SEM (*n* = 6). ^a^*p* < 0.05: significant compared with the normal group. ^b^*p* < 0.05: significant compared with the paclitaxel-administered group. Percentage changes were calculated by comparing the paclitaxel-administered group with the normal and the paclitaxel-administered groups treated with naringin and/or naringenin with the paclitaxel-administered group.

**Table 2:** Effect of naringin and/or naringenin on serum parameters related to heart function.

Parameters and groups	CK-MB(U/L)	% change	LDH (U/L)	% change
Normal	8.42 ± 0.71	—	586.75 ± 36.85	—
Paclitaxel	38.67 ± 4.41^a^	359.26	2309.17 ± 105.09^a^	293.55
Paclitaxel + naringin	20.83 ± 1.72^ab^	**−**46.13	1237.50 ± 152.19^ab^	**−**46.41
Paclitaxel + naringenin	17.20 ± 1.05^b^	**−**55.52	1180.83 ± 105.25^ab^	**−**48.86
Paclitaxel + naringin + naringenin	20.20 ± 1.54^ab^	**−**47.76	1135.83 ± 48.25^ab^	**−**50.81

Data are expressed as mean ± SEM (n = 6). a *p* < 0.05: significant compared with normal group. b *p* < 0.05: significant compared with paclitaxel-administered group. Percentage changes were calculated by comparing paclitaxel-administered group with normal, and paclitaxel-administered groups treated with naringin and/or naringenin with paclitaxel-administered group.

**Table 3:** Effect of naringin and/or naringenin on kidney LPO, GSH content, and SOD and GPx activities.

Parameters and groups	LPO (nmol MDA/100 mg tissue/hour)	% change	GSH (nmol/100 mg tissue)	% change	SOD (U/g)	% change	GPx (mU/100 mg tissue)	% change
Normal	14.20 ± 0.83	—	108.12 ± 3.32	—	18.93 ± 0 .19	—	104.16 ± 1.12	—
Paclitaxel	22.00 ± 0.93^a^	54.93	50.7 ± 3.95^a^	**−**53.09	17.38 ± 0.20^a^	**−**8.19	79.962.18^a^	**−**23.23
Paclitaxel + naringin	14.80 ± 0.81^b^	**−**32.73	96.22 ± 3.77^b^	89.74	18.48 ± 0.11^b^	6.33	91.96 ± 1.43^ab^	15.01
Paclitaxel + naringenin	17.40 ± 0.51^b^	**−**20.91	89.95 ± 4.20^ab^	77.38	18.59 ± 0.14^b^	6.96	88.45 ± 0.93^ab^	10.62
Paclitaxel + naringin + naringenin	16.20 ± 1.3^b^	**−**26.36	92.42 ± 3.37^ab^	82.25	18.62 ± 0.23^b^	7.13	86.72 ± 2.69^a^	8.45

Data are expressed as mean ± SEM (n = 6). a *p* < 0.05: significant compared with normal group. b *p* < 0.05: significant compared with paclitaxel-administered group. Percentage changes were calculated by comparing paclitaxel-administered group with normal, and paclitaxel-administered groups treated with naringin and/or naringenin with paclitaxel-administered group.

**Table 4:** Effect of naringin and/or naringenin on heart LPO, GSH content, and SOD and GPx activities.

Parameters and groups	LPO (nmol MDA/100 mg tissue/hour)	% change	GSH (nmol/100 mg tissue)	% change	SOD (U/g)	% change	GPx (mU/100 mg tissue)	% change
Normal	11.90 ± 0.67	—	89.30 ± 3.30	—	18.82 ± 0.04	—	100.90 ± 1.60	—
Paclitaxel	22.40 ± 0.63^a^	88.24	53.60 ± 2.90^a^	**−**40	17.05 ± 0.19^a^	**−**9.40	86.40 ± 1.70^a^	**−**14.37
Paclitaxel + naringin	12.50 ± 0.98^b^	**−**44.20	71.40 ± 1.40^ab^	33.21	18.47 ± 0.08^b^	8.32	98.20 ± 0.70^b^	13.66
Paclitaxel + naringenin	12.90 ± 0.79^b^	**−**42.41	63.50 ± 4.20^a^	18.47	18.38 ± 0.06^ab^	7.80	92.20 ± 0.30^ab^	6.71
Paclitaxel + naringin + naringenin	16.80 ± 0.15^ab^	**−**25.00	86.20±0.80^b^	60.82	18.36 ± 0.04^ab^	7.68	95.50 ± 1.40^ab^	10.53

Data are expressed as mean ± SEM (n = 6). a *p* < 0.05: significant compared with normal group. b *p* < 0.05: significant compared with paclitaxel-administered group. Percentage changes were calculated by comparing paclitaxel-administered group with normal, and paclitaxel-administered groups treated with naringin and/or naringenin with paclitaxel-administered group.

**Table 5:** Pathological renal lesion scores in different groups.

Parameters and groups	Degenerative of renal tubules	Necrosis of renal tubules	Congestion	Leukocyte infiltration	Glomerulonephritis	Apoptosis
Normal	−	−	−	−	−	−
Paclitaxel	+++	++	+++	+++	+++	++++
Paclitaxel + naringin	++	++	++	++	++	++
Paclitaxel + naringenin	++	+	++	−	+	+
Paclitaxel + naringin + naringenin	+	−	+	−	−	+

Lesion types are (−) absence, (+) minimal, (++) mild, (+++) moderate, and (++++) severe.

**Table 6:** Pathological cardiac lesion scores in different groups.

Parameters and groups	Coagulative necrosis (hyalinosis)	Leukocyte infiltration	Apoptosis
Normal	−	−	**−**
Paclitaxel	++	+++	**++**
Paclitaxel + naringin	+	−	**+**
Paclitaxel + naringenin	++	+	**−**
Paclitaxel + naringin + naringenin	+	+	**−**

Lesion types are (−) absence, (+) minimal, (++) mild, (+++) moderate, and (++++) severe.

## Data Availability

All data are available from the corresponding author upon reasonable request.
